The article "Reform of PBL Teaching Mode of Microcomputer System and Embedded Application Course Group" was retracted in 2023. Reasons: signs of a paper mill; suspected computer-generated content; unreliable results or conclusions; concerns about the data.

# Reform of PBL Teaching Mode of Microcomputer System and Embedded Application Course Group

**DOI:** 10.1155/2022/5396393

**Published:** 2022-04-23

**Authors:** Peifen Ding, Baoqi Zhao

**Affiliations:** ^1^School of Economics and Management, Zhejiang Business Technology Institute, Ningbo 315012, Zhejiang, China; ^2^School of Electronic Information Engineering, Ningbo Polytechnic, Ningbo 315800, China

## Abstract

In recent years, the problem-based learning (PBL) model has become a hot spot in the education field. Its unique “learner”-centered and “problem-based” characteristics have been widely used in teaching. Make a useful attempt to comply with the development of the times and the requirements of education. This article puts forward the research on the reform of PBL teaching mode based on the microcomputer system and embedded application course group, using literature data method, fuzzy comprehensive analysis method, questionnaire survey method and other methods to explore. This paper designs the experiment of PBL teaching mode reform based on the microcomputer system and embedded application course group, analyzes the domestic research status of PBL teaching mode, and analyzes and summarizes the teaching effect of PBL. The average score of the experimental class with PBL teaching was 74.76 points, and the passing rate reached 95.13%; while the average score of the control group was 70.21 points, and the passing rate was 92.30%. The PBL teaching model of the microcomputer system and embedded application course group conforms to the general direction of my country's education development and reform. It can cultivate students' innovative consciousness and problem-solving ability. It has a certain reference value for improving the quality of course teaching and also provides teachers with a Kind of new teaching ideas and approaches.

## 1. Introduction

Now most universities and schools continue to use the old embedded system experimental teaching and education system, but the effect is not obvious. First of all, regarding the arrangement of experiments, there are many single basic experiments, few comprehensive development experiments, and insufficient systematic experiments. In addition, previous experimental education always conducted experiments in the order of related courses. Although this method is conducive to consolidating the theory of teaching courses, it is difficult for students to intuitively and comprehensively understand the design of the entire experimental system through experiments because there is no correlation between various experiments. Therefore, reforming the teaching mode of embedded application courses is the most important task at present.

The article "Reform of PBL Teaching Mode of Microcomputer System and Embedded Application Course Group" was retracted in 2023. Reasons: signs of a paper mill; suspected computer-generated content; unreliable results or conclusions; concerns about the data.

In addition to focusing on theory, the microcomputer system and embedded application course also emphasizes the practicality of the course. In the education links of theory, experiment, curriculum design, etc., they have higher requirements for theoretical knowledge and practical ability. According to these requirements, circuit design, software programming and system error detection can be completed systematically. Traditional teaching methods cannot stimulate students' possibilities, and it is difficult to use various forms to enable students to communicate and learn more intuitively and deeply. Therefore, the implementation of microcomputer system and embedded PBL teaching reform is a good way to improve students' learning ability.

The PBL teaching mode of the microcomputer system and embedded application course group is in line with the general direction of China's education development and reform. Studying and applying this teaching mode can cultivate students' innovative consciousness and problem-solving ability. This has a certain reference value for improving the quality of course teaching, and also provides a new teaching idea and method for teachers.

Alrahlah's article aims to explore the effectiveness of problem-based learning (PBL) as a dental teaching method. PBL was developed more than 40 years ago in response to the problems and limitations of traditional teaching methods. This article reviews several aspects of PBL teaching method and discusses the reasons why PBL teaching method plays an important role in dental education. There is evidence that compared with traditional teaching methods, students in PBL courses show higher professional skills and effective learning. Because the PBL teaching method is student-centered and problem-based, students obtain methods and answers to solve problems through discussion, research and other methods, which makes students' learning change from passive to active, from blind to purposeful The search for answers to questions and the active exploration process of substance. However, his experimental process is not rigorous, and the number of experimental samples is very small [1]. Rodriguez-Sanchez MC This article presents a case study that analyzes project-based learning (PBL) combined with collaborative learning (CL) and industry best practices, combined with information and communication technology, open source software and open source hardware tools, in dedicated microcontrollers and The pros and cons of an engineering master's program used in embedded systems. In addition to meeting industry requirements in content and methods, this course also cultivates students' abilities in problem solving, independent study, teamwork and technical knowledge. Since the PBL method itself does not ensure teamwork, it is complemented by CL. Design review meetings (as described in IEC 61160), deliverables and organizational resources are also introduced to reflect industry needs. This structure (The structure is a combination of Project-Based Learning (PBL) with Collaborative Learning (CL) and industry best practices, combining ICT, open source software and open source hardware tools for the structure of specialized microcontrollers and embedded systems) integrates course content and student academic performance in a simulated industrial environment. This course allows students to build a modular household appliance management system and implement control software. However, his research and analysis are not clear and complete enough, so additional research is needed [2]. Osamnia M proposes a new automatic course generation system in this research, which is embedded in the online lecture platform to establish the electronic course content of higher education online lectures. The purpose of the system is based on a series of events, real-time and automatic synchronization of the speaker's video stream and presentation slides, thereby speeding up the development of electronic content. The system detects events that occur during the online lecture, such as slide changes, cursor positioning, and video quality changes, and links them to the exact location of the recorded video stream, so that they are displayed in the real presentation. The system implements a writing algorithm, the Curriculum Generation (CG) algorithm, which realizes a fast and fully automatic writing process. In addition, the created content is integrated into a web-based learning environment, which is an important step in the long road to make learning a more independent concept of time and space, everything about the Internet (IoE) education. The paper also introduces the actual application of the system and illustrates the practicability and effectiveness of the system. However, during his embedded online teaching process, many equipment problems appeared, which have not been solved yet [3].

The article "Reform of PBL Teaching Mode of Microcomputer System and Embedded Application Course Group" was retracted in 2023. Reasons: signs of a paper mill; suspected computer-generated content; unreliable results or conclusions; concerns about the data.

The innovations of this article are: (1) using a variety of methods for analysis: literature data method, fuzzy synthesis method (Fuzzy comprehensive evaluation method is a comprehensive evaluation method based on fuzzy mathematics. The comprehensive evaluation method transforms qualitative evaluation into quantitative evaluation according to the membership degree theory of fuzzy mathematics, that is, using fuzzy mathematics to make a general evaluation of things or objects restricted by many factors. It has the characteristics of clear results and strong systematicness, which can better solve vague and difficult-to-quantify problems, and is suitable for solving various non-deterministic problems.), questionnaire survey method, etc., through these methods to discuss the relevant research results of the sports industry from the theoretical perspective; (2) qualitative research combines with quantitative research and fully analyzes the research data; (3) the pioneering reform of the microcomputer system and the embedded application to the teaching mode improves the teaching quality and provides new teaching ideas and methods.

## 2. The PBL Teaching Mode Reform Method of the Microcomputer System and Embedded Application Course Group

### 2.1. Embedded Application System

Embedded system technology is the most popular technology today, and its scope of application far exceeds other types of general-purpose computers [4]. In order to learn, research and use embedded technology, many domestic universities plan to develop embedded application teaching, aiming to change the current teaching dilemma and have a new breakthrough in education and teaching [5].

The essence of the embedded system is to deploy various necessary software and hardware facilities with the assistance of the computer system. At the same time, it is a special computer system with high requirements for its function, size, power consumption and other high standards with the application as the center [6, 7]. The scope of its objects includes almost all electrical equipment around us, such as televisions, notebooks, portable computers, multimedia equipment, medical equipment, and even switches [1].

The types of embedded systems are different, and their characteristics are also different, most of which are derived from its basic elements [8]. The basic elements of embedded system are embeddedness, speciality and computer system. Embedding means to embed software into Flash memory, speciality refers to a specific application field and occasion, tailor-made special-purpose system suitable for the occasion, computer system means that it must have the composition of the computer system, which is a computer system. (1) User-oriented, product-oriented, and application-oriented. Unlike general-purpose computers, energy consumption, size, cost, reliability, speed, processing power, electromagnetic compatibility, etc. are restricted by application requirements [9]. If they are independent from the application, they will lose effectiveness. (2) The system is streamlined. (3) High efficiency and high reliability [10]. (4) Relative stability. (5) Special development tools and environment.

The article "Reform of PBL Teaching Mode of Microcomputer System and Embedded Application Course Group" was retracted in 2023. Reasons: signs of a paper mill; suspected computer-generated content; unreliable results or conclusions; concerns about the data.

With the rapid development of information technology based on computer, Internet and communication technology, embedded system development technology has also achieved rapid development [11]. As a special computer system, embedded system is becoming more and more important in the Internet era, and its application range is more and more extensive, especially in the field of education [12].

The embedded system has the following characteristics when applied to teaching: comprehensiveness. This includes many micro-systems such as electronic equipment, computers, and automatic control [13]. It is very comprehensive and can include courses such as microcomputer principles, electronic circuit technology, single-brand microcomputer design, operating systems, etc. It is a perfect combination of software and hardware equipment. It can be used as a basic platform course for large enterprises, such as computers, power electronics, automatic control, etc. [14]. Experiments are an important part of embedded system teaching.

The application of embedded systems in teaching can make full use of the existing equipment in the computer room, reduce the hardware maintenance of experimental equipment, and be close to the actual engineering system, narrowing the distance between learning and employment. Practice has proved that this embedded system The teaching method can not only reduce the cost and has obvious economic advantages, but also has a high promotion value.

### 2.2. PBL Teaching Mode

PBL is the abbreviation of Problem-based Learning. So far, there has not been a unified understanding of the definition of PBL. However, the most commonly accepted concept of PBL is as follows: PBL is a teaching method that puts learning under the actual problem situation, through the cooperation of teachers and students in teams, joint exploration, and discovering and solving problems together [15, 16]. The purpose of the PBL teaching model can be summarized in one sentence: through the entire learning activities of PBL, students' interest in learning is stimulated, and students' multiple abilities can be improved and developed [17].

The elements of PBL boil down to the problem situation, students and teachers. The author believes that among the three elements, the core is the problem situation, which is the driving force that triggers students to think about solving problems; students are the main part, who understand the problem with the consciousness of “master,” discover the problem, and finally solve the problem; the teacher is the whole process Instructor, to promote students to solve problems [14, 18].

From the beginning of the 20th century to the present, many modern learning theories and educational concepts have revealed the essence of human learning, such as multiple intelligence theory, constructivism theory, quality education and the concept of simultaneous knowledge and action, etc. [19]. People's intelligence is embodied in ability, and intelligence is formed and developed through the mastery of knowledge. Without the activities of mastering knowledge, our intelligence cannot be expressed or developed, and the difficulty and speed of mastering knowledge, It also depends on the level of intellectual development. Intelligence provides favorable conditions for the acquisition of knowledge, and the acquisition of knowledge further promotes the development of intelligence. PBL teaching reform has found certain theoretical support from these learning theories.

The article "Reform of PBL Teaching Mode of Microcomputer System and Embedded Application Course Group" was retracted in 2023. Reasons: signs of a paper mill; suspected computer-generated content; unreliable results or conclusions; concerns about the data.

#### 2.2.1. Constructivist Theory

Among the many educational theories at home and abroad, constructivist learning theory has always occupied the mainstream position, and has been unanimously praised by experts and scholars in the education field. The constructivist learning theory was first proposed by Piaget, and he is also the most representative figure, who has made the most outstanding contribution to constructivism. Later, after Vygotsky, Ausubel and other experts enriched and perfected the content of constructivism, the theoretical system of constructivism became mature step by step [20].

Constructivist learning theory believes that knowledge is not transmitted to students by teachers in the form of indirect experience, but students are constructed through active meaning. There are four most important aspects in constructivist theory, namely, context, cooperation, communication, and meaning construction [21, 22]. In detail, it can be understood that in the process of active construction, a student first needs to create a reasonable situation and understand the corresponding cultural background; second, to cooperate with others, communicate, and obtain more relevant information through communication Information, or get some help, etc. Finally, it is the realization of the above steps that can form a meaningful construction, highlighting its contextuality, interaction and knowledge dynamics [23].

Context: helps to establish the subjective meaning of students. In addition, it is also very important to use PBL to create a problem environment. Cooperation: through the entire learning process, the discovery and analysis of problems, the collection and processing of learning resources, the mutual assistance between teachers and students, and the evaluation of learning results must be carried out through cooperation. Communication: this is a necessary part of the learning activity. In the process of cooperation, students must speak. Only through communication and dialogue can they reach the ultimate goal of solving the problem. Meaning construction: it is the ultimate goal of learning activities. The process of students completing meaning construction is actually the process of integrating and processing knowledge, and it is also a process from shallow understanding to deep understanding. The main body of the PBL teaching model is students. It is problem- and project-oriented learning and emphasizes students' autonomous learning and active inquiry learning.

The article "Reform of PBL Teaching Mode of Microcomputer System and Embedded Application Course Group" was retracted in 2023. Reasons: signs of a paper mill; suspected computer-generated content; unreliable results or conclusions; concerns about the data.

#### 2.2.2. Multiple Intelligence Theory

In the 1980s, American psychology professor Howard Gardner proposed the theory of multiple intelligences. He believes that intelligence is not only based on language, logic and mathematics. In addition to the above factors, there are more different combinations that determine the differences between people and each person's ability.

The concept of talents advocated by the theory of multiple intelligences is the concept of comprehensive and diversified development of people, not the narrow concept of talents in the traditional sense. It emphasizes that everyone has different potentials. As long as they are properly educated, students' potentials can be developed and become talents in a certain area. However, traditional education overemphasizes speech-language intelligence, logic-mathematics intelligence, and relying solely on a piece of paper and a pen determines the intelligence of students, thus ignoring the potential of students in other areas, and inhibiting the cultivation of talents. Development is very one-sided. Regarding school education, Gardner believes that problem-based learning can use language and language intelligence to change traditional knowledge theories. With logic and mathematics knowledge as the core, schools and teachers are encouraged to develop each student's strengths and personality points. The problem-based learning model is to create problem situations, with students as the main body, giving students more space, allowing students to independently explore problems according to their own hobbies and specialties, participate in discussion of problems, and teachers can integrate multiple intelligences into teaching in a targeted manner In order to improve students' multiple intelligence.

#### 2.2.3. The Concept of Quality Education and Knowledge and Action Simultaneously

Quality education is based on the needs of the overall development of society and mankind, with the first goal of improving the basic comprehensive quality of students, actively supporting the spirit of running a school with students as the main body, and focusing on development. Develop students' possibility, personality formation and innovative practical ability. Its connotation can be understood as: two needs: the needs of sustainable social development and the needs of all-round human development; three developments: all-round development, overall development, and individual development; two focus: focus on the development of students' potential and focus on student innovation And the cultivation of practical ability; an operational spirit: to vigorously advocate and implement subjective education. The concept of quality education has become synonymous with the concept of modern education and is a collection of ideal education concepts based on the overall development needs of society and mankind. In recent years, the concept of Zhineng curriculum has focused on the “ability-based” in the positioning of curriculum functions, and required “knowledge and action” in the selection of curriculum learning content. The organization of curriculum content is based on “learners” and emphasizes the content of the curriculum. The system should integrate all ideological and action, with “professional adaptability training” as the core goal, and the “problem-based teaching materials” put forward in the knowledge-ability curriculum is consistent with the PBL's “problem-driven” concept. The educational goal of PBL is to cultivate students' problem thinking and teamwork spirit, and master the ability of independent learning and problem solving. This is consistent with the concept of quality education and knowledge courses. The construction and practice of PBL teaching mode under the guidance of these two theoretical ideas conform to the development of the times.  Figure 1 shows the PBL teaching class.

The article "Reform of PBL Teaching Mode of Microcomputer System and Embedded Application Course Group" was retracted in 2023. Reasons: signs of a paper mill; suspected computer-generated content; unreliable results or conclusions; concerns about the data.

From the above analysis, it can be seen that on the basis of these theories, modern education models need to consciously adapt to the needs of society and human development, and more need to pay attention to the development and improvement of students' in-depth thinking and practical skills, and pay attention to teachers in the process of teaching activities. Guidance, the subjectivity of students and the interaction and collaboration between teachers and students, grasp the integrity of teaching objectives, focus on changing the learning methods of traditional teaching, and create an ideal classroom atmosphere and teaching form. This puts forward higher requirements for the PBL teaching model, and it is necessary to guide the teaching reform from the roles of teachers and students, teaching methods, teaching environment and teaching evaluation. In addition to the basic teaching knowledge of blackboard writing in the classroom, it is also necessary to have a certain knowledge of the Internet, computer knowledge and the use of computers, the use of computer systems and other aspects of knowledge.

Constructivist learning theory has always occupied the mainstream position and has been unanimously recognized by experts and scholars in the education field; the theory of multiple intelligences emphasizes that everyone has different potentials, and as long as they are properly educated, everyone's potential can be developed; quality education requires both knowledge and action The concept emphasizes quality education and behavior training.

### 2.3. Teaching Evaluation Methods

As a standard comprehensive evaluation method, the fuzzy comprehensive evaluation method comes from fuzzy mathematics that converts qualitative evaluation into quantitative evaluation. The evaluation results must be suitable for nonquantitative evaluation results. The evaluation of teaching effects using this method often has clear and systematic characteristics. The most notable feature of the fuzzy comprehensive evaluation method is: take the optimal evaluation factor as the benchmark, and its evaluation value is 1; It can determine the functional relationship between the evaluation value and the evaluation factor value (ie: membership function) according to the characteristics of various evaluation factors. There are many ways to determine this functional relationship (membership function), for example, F statistics methods, various types of F distributions, etc. Of course, experienced bid evaluation experts can also be invited to evaluate and give the evaluation value directly.

Definition of fuzzy set: assuming as a domain, a mapping to the interval can determine a fuzzy subset of the domain. The fuzzy set on the universe is generally expressed as

(1) $$\begin{array}{c} M=\left\{\frac{\mu_{M}\left(\mu_{1}\right)}{\mu_{1}},\frac{\mu_{2}\left(\mu_{2}\right)}{\mu_{2}},\frac{\mu_{M}\left(\mu_{3}\right)}{\mu_{3}}\cdots \right\}. \end{array}$$

For many finite domains, the fuzzy set can be expressed as follows:

(2) $$\begin{array}{c} M=\left(\mu_{M}\left(\mu_{1}\right),\mu_{M}\left(\mu_{2}\right),\ldots ,\mu_{M}\left(\mu_{n}\right)\right). \end{array}$$

Membership function is a very important concept in fuzzy mathematics. The specific expression is

(3) $$\begin{array}{c} \mu_{M}\left(x\right)=\left\{\begin{array}{c} 1,x\in M\\ 0<\mu_{M}\left(x\right)<1\\ 0,x\notin M \end{array}.\right. \end{array}$$

The fuzzy comprehensive evaluation method is based on the in-depth application of the fuzzy transformation principle, fully considering the influence and evaluation of various factors on different aspects. Therefore, the basic principle is based on the correlation between the evaluation object and the weight of each evaluation index, the evaluation set of various levels from good to bad, and the promotion of multiple factors to carry out fuzzy evaluation corresponding to each index.

The article "Reform of PBL Teaching Mode of Microcomputer System and Embedded Application Course Group" was retracted in 2023. Reasons: signs of a paper mill; suspected computer-generated content; unreliable results or conclusions; concerns about the data.

The main calculation formula of fuzzy transformation is

(4) $$\begin{array}{c} \beta_{j}=\vee \left(a_{i}\wedge r_{ij}\right)\left(j=1,2,3,\ldots ,m\right). \end{array}$$

The specific calculation formula for multiplying instead of taking the small method is as follows:

(5) $$\begin{array}{c} \beta_{j}=\vee \left(a_{i}r_{ij}\right)\left(j=1,2,3,\ldots ,m\right). \end{array}$$

Similarly, the specific calculation formula for adding instead of taking the larger is

(6) $$\begin{array}{c} \beta_{j}=\sum_{i=1}^{n}\left(a_{i}\wedge r_{ij}\right)\left(j=1,2,3,\ldots ,m\right). \end{array}$$

The calculation formula of the weighted average i

(7) $$\begin{array}{c} \chi_{j}=\sum_{i=1}^{n}\left(a_{i}r_{ij}\right)\left(j=1,2,3\ldots ,m\right). \end{array}$$

This is a method of calculating the weighted vector based on the multiplication of the general matrix. It realizes the multiplication of the required evaluation matrix and uses the weighted average algorithm to evaluate the effect of all the elements contained in the result, which has a strong comprehensiveness.

Arrange all the values participating in the evaluation in a matrix, the matrix form is

(8) $$\begin{array}{c} M={\left(a_{ij}\right)}_{m\times n}\left[\begin{array}{cccc} \frac{a_{1}}{a_{1}} & \frac{a_{1}}{a_{2}} & \cdots & \frac{a_{1}}{a_{n}}\\ \frac{a_{2}}{a_{1}} & \frac{a_{2}}{a_{2}} & \cdots & \frac{a_{2}}{a_{n}}\\ \vdots & \vdots & \ddots & \vdots \\ \frac{a_{n}}{a_{1}} & \frac{a_{n}}{a_{2}} & \cdots & \frac{a_{n}}{a_{n}} \end{array}\right]. \end{array}$$

After the above judgment matrix is constructed, combined with the n evaluation indicators that have been determined, the weight of each indicator can be determined by calculating the maximum eigenvalue of the judgment matrix, and the corresponding eigenvector can be obtained, which can further determine the value of each indicator. The relative weight is determined, and the detailed process is as follows: First, calculate the geometric average of all elements of the judgment matrix, as shown in the following formula.

(9) $$\begin{array}{c} \varpi_{i}=\sqrt[{n}]{\prod_{j=1}^{n}a_{ij}\left(j=1,2,\ldots ,n\right)}. \end{array}$$

The above geometric mean value is normalized, and the specific formula is shown in the formula.

(10) $$\begin{array}{c} \omega_{i}=\frac{\varpi_{i}}{\sum_{i=1}^{n}\varpi_{i}\left(i=1,2,\ldots ,n\right)}. \end{array}$$

The comprehensive evaluation matrix is

(11) $$\begin{array}{c} Q=\left[\begin{array}{cccc} r_{11} & r_{12} & \cdots & r_{1m}\\ r_{21} & r_{22} & \cdots & r_{2m}\\ r_{31} & r_{32} & \cdots & r_{3m}\\ \vdots & \vdots & \ddots & \vdots \\ r_{m1} & r_{m2} & \ldots & r_{km} \end{array}\right]. \end{array}$$

The assignment matrix is

(12) $$\begin{array}{c} G=\left[\begin{array}{c} g_{1}\\ g_{2}\\ \vdots \\ g_{M} \end{array}\right], \end{array}$$

then,

(13) $$\begin{array}{c} X=Q\cdot G=\left(\frac{b_{1}}{\sum b_{1}},\frac{b_{2}}{\sum b_{2}},\ldots ,\frac{b_{m}}{\sum b_{j}}\right)\left[\begin{array}{c} g_{1}\\ g_{2}\\ \vdots \\ g_{M} \end{array}\right]. \end{array}$$

X represents the score obtained from the comprehensive evaluation of the evaluation object.

The article "Reform of PBL Teaching Mode of Microcomputer System and Embedded Application Course Group" was retracted in 2023. Reasons: signs of a paper mill; suspected computer-generated content; unreliable results or conclusions; concerns about the data.

On the basis of the above matrix, a single-layer comprehensive evaluation matrix is obtained as follows:

(14) $$\begin{array}{c} P=Q*R=\left(W_{1},W_{2},\cdots ,W_{N}\right)*\left[\begin{array}{cccc} r_{11} & r_{12} & \cdots & r_{1m}\\ r_{21} & r_{22} & \cdots & r_{2m}\\ r_{31} & r_{32} & \cdots & r_{3m}\\ \vdots & \vdots & \ddots & \vdots \\ r_{m1} & r_{m2} & \cdots & r_{mn} \end{array}\right]. \end{array}$$

The weight coefficient is

(15) $$\begin{array}{c} E=\frac{\lambda_{1}x_{1}+\lambda_{2}x_{c}+\cdots +\lambda_{k}x_{k}}{\sum_{i=1}^{p}\lambda_{i}}. \end{array}$$

## 3. PBL Teaching Mode Reform Experiment of Microcomputer System and Embedded Application Course Group

A good teaching model is a necessary condition for teaching. PBL-based teaching model reform is a key factor that affects the teaching effect, and teaching design is also an important link that affects the teaching effect. The PBL teaching model reform experiment of the microcomputer system and embedded application course group carried out in this paper. The selected research object is a third-year computer major in a university. Taking the programming course as an example, the teaching objectives, learner characteristics, learning content, learning Environment, teaching strategy, teaching evaluation and many other factors carry out PBL teaching design for programming courses. The experimental process is to analyze the current situation of the teaching model, put forward the corresponding problems, then investigate a questionnaire for these problems, and then analyze the PBL teaching model introduced in this paper, calculate the application, get the students and teachers to score the teaching model, and get the final test results.

### 3.1. Determine the Teaching Goal

PBL education goals play an important role in teaching, education evaluation and motivation derivation. The scientific rationality of educational goals plays a very important role in the smooth implementation of PBL teaching mode. The educational goals of PBL can be divided into knowledge goals, skill goals, and emotional goals.

The article "Reform of PBL Teaching Mode of Microcomputer System and Embedded Application Course Group" was retracted in 2023. Reasons: signs of a paper mill; suspected computer-generated content; unreliable results or conclusions; concerns about the data.

The design of knowledge goals: In PBL teaching, the design of knowledge goals is very important and requires a certain degree of difficulty. When formulating a plan, it is necessary to consider the context of knowledge learning and the problem as well as the method of closely integrating learning topics based on the textbook, and plan those that focus on the scope and depth of knowledge adjustment, diversity and specificity, application and understanding. The design of skill objectives: the ability of obtaining information, analyzing and evaluating students in PBL, as well as the ability to find and solve problems. The main purpose is to cultivate students' cooperation and autonomous learning ability, and improve students' awareness of active learning. Design emotional goals: Emotions are positive or negative psychological responses to external stimuli. The educational goals in the emotional field are divided into five levels: acceptance, response, value, organization, and personalization according to the degree of internalization of value.

### 3.2. Experimental Content

PBL is a kind of problem-based learning. It is a learning method that allows students to actively discover and solve problems. Its starting point is the development of students, which shows that the essence of PBL belongs to the category of “learning.” But from the perspective of teaching, only by starting with “teaching” can the effectiveness of PBL be truly guaranteed. The biggest difference between PBL's teaching activities and traditional classroom teaching is that it is open, spends more time, and breaks through the limitations of time and space. In the whole teaching activities, teachers provide appropriate and effective guidance, which has a great influence on the quality of teaching.

#### 3.2.1. Problem Teaching Strategy

The smooth development of the entire teaching process is inseparable from teachers' effective guidance and moderate participation. Teachers should pay attention to the following points in the PBL teaching strategy. (1) Focus on cultivating students' problem awareness. In the past teaching, teachers used how much knowledge the students learned to measure the level of learning ability. In PBL teaching activities, teachers should let students discover and solve problems proactively, which is also the teaching goal of PBL. Therefore, teachers should change their ideology and focus on cultivating students' problem awareness. Choose real questions and guide students to ask questions. Determine the problem, combine subject knowledge with social development, and combine students' interests and expertise. (2) PBL training. The students just started to come into contact with the PBL teaching mode. They are not very familiar with it and lack experience, and the subjectivity of learning is not strong. A PBL training process is needed to teach students the corresponding learning methods to ensure the smooth development of PBL. In this stage, teachers should tell students some background experience of PBL, including its nature, learning and operation methods, etc. Through training, let students have a macro-perceptual understanding of the background experience of PBL teaching.

The article "Reform of PBL Teaching Mode of Microcomputer System and Embedded Application Course Group" was retracted in 2023. Reasons: signs of a paper mill; suspected computer-generated content; unreliable results or conclusions; concerns about the data.

#### 3.2.2. Methodological Guidance Strategy

This time, the teaching design of PBL in the program design course, although the research object is juniors, they already have a high level of thinking, but they do not know much about PBL, lack experience in it, and their thinking is still stuck. In order to make teaching start smoothly, teachers should provide guidance in many ways. (1) Students change their learning concepts. In PBL teaching activities, students are the “masters” of learning, and teachers should guide students to change their concepts, take the initiative to acquire knowledge, and play the role of learning subjects.

(2) Introduction of relevant knowledge background. In PBL teaching, the problem design is generally more complicated, and teachers need to introduce the knowledge background of the problem. In this process, teachers not only provide students with the knowledge needed in the problem, but also teach students how to learn, otherwise the value of PBL will be lost. (3) Change of thinking mode. In PBL, teachers and students must change their way of thinking. Don't stick to traditional teaching ideas. As long as you learn the rules and regulations in the book, you can achieve the goal. Teachers and students should stand at a higher height and learn to analyze problems from multiple angles., Solve the problem.

### 3.3. Experimental Method

The research of this thesis mainly adopts literature research method, questionnaire method, action research method, case analysis method and evaluation research method. (1) Literature research method. Check the literature related to the PBL teaching model to understand the latest research results at home and abroad. First of all, by searching the relevant literature of major domestic academic journals on the China Knowledge Network (CNKI) with “problem-based learning/PBL” as the key word, we have a clear understanding of the research development trend of PBL, which is useful for research. Get ready for it in depth. The second is to use the Internet, books and other channels to obtain documents related to this research. (2) Questionnaire method. Designing questionnaires, preexperiment test questionnaires to understand the learning attitude and cognitive level of the experimental class students; postexperiment test questionnaires to investigate the teaching situation of the experimental class, understand the implementation of PBL, to verify the teaching effect. (3) Action research method. This is the main research method of this subject. Follow-up survey visits to teachers and students in a certain university will provide effective cases and arguments for research. (4) Case analysis method. Case analysis is the process of looking at the essential structure through the phenomenon of individual cases. According to the purpose of the research, by cooperating with the teacher, taking the university programming course as an example, carry out the specific application of PBL teaching mode in the classroom, form a case, and then analyze and summarize the experience. (5) Fuzzy comprehensive evaluation method. The teaching effect of PBL class and ordinary class is compared, data analysis is carried out, and practice results are verified. This method is often used.

The article "Reform of PBL Teaching Mode of Microcomputer System and Embedded Application Course Group" was retracted in 2023. Reasons: signs of a paper mill; suspected computer-generated content; unreliable results or conclusions; concerns about the data.

### 3.4. Experimental Evaluation

Different from the traditional teaching model, the roles of teachers and students in PBL have changed. Teachers become the “instructors” of learning, and students become the “main body” of learning, so the evaluation method has also changed. Therefore, in the PBL evaluation method, self-evaluation, mutual evaluation and teacher evaluation are generally used organically, with process evaluation as the main and summative evaluation as the supplement.

(1) Self-evaluation allows students to think in more detail about what they already know and what they do not know, as well as what they should know to complete a given learning task, so that students can clarify the lack of knowledge in order to promote more meaningful learning. Through student self-evaluation, students can evaluate their own performance, know themselves, check for deficiencies and make up for omissions, so that students have more opportunities to think deeply about their own deficiencies, and at the same time teachers can understand students' self-feelings. (2) Mutual evaluation is the evaluation between peers, which is to let other members of the group evaluate the students personally, evaluate the enthusiasm and initiative of the students in the group to participate in problem solving, etc., and highlight the group cooperative learning. Since we have to cooperate with others in real life, mutual evaluation is a feasible method to detect the growth of students. This process emphasizes the importance of cooperation in the PBL environment. (3) Teacher evaluation is the evaluation of individual students by teachers, and the investigation of students' performance in the entire PBL learning process. Compared with students' self-evaluation and mutual evaluation, teacher evaluation focuses on students' performance and participation in the activity process, which is a relatively objective evaluation. The feedback provided by teachers should encourage students to explore and help students to learn better and deeper.

The article "Reform of PBL Teaching Mode of Microcomputer System and Embedded Application Course Group" was retracted in 2023. Reasons: signs of a paper mill; suspected computer-generated content; unreliable results or conclusions; concerns about the data.

Figure 2 is the basic flow chart of PBL teaching mode.

## 4. Reform of PBL Computer Systems and Embedded Applications Course Group Analysis

### 4.1. Background Analysis of PBL Teaching Mode

In our country, the PBL teaching model started relatively late. In the 1980s, PBL was introduced into the medical field; in the 1990s, PBL has been tried out in some courses by universities such as Hunan Medical University, and the teaching effect achieved is better than traditional education methods, and it can improve students' innovation and practice. The ability to solve problems, but there are still some limitations. Like the pattern of foreign PBL development, PBL also extends from the field of medical education to more other fields, such as trying to apply it in courses such as mathematics and computer.

In order to understand the current status of the research on the number of documents on the domestic PBL teaching model, this paper selects the period from 2008 to 2018 as the time limit, selects “PBL” as the search term, selects “teaching model” as the search topic, and retrieves the full-text database of Chinese journals And the excellent thesis database, the search results show that a total of 1,692 papers have been published in China, including 1,494 papers, 4 doctoral theses, and 194 master's theses. As shown in Table 1 and Figure 3, this article compares the publication year of books and periodicals and the number of documents to form the distribution of the number of documents in the PBL teaching model reform.

Aiming at the application of PBL in the teaching practice of Chinese universities and vocational technical colleges, combined with the development status of my country's microcomputer system and embedded application courses, the introduction of PBL teaching into such courses will greatly reverse the current teaching of embedded courses. The status quo, changing the old training mode, provides a new idea for the development of microcomputer systems and embedded courses.

From the data in Table 2 and Figure 4, it can be seen that 2.63% of students said they knew PBL very well, 5.26% of students said they knew, 21.05% of students said they knew a little bit, and 71.05% of students said they had never heard of it. Regarding the issue of having carried out PBL in previous courses, 5.26% of the students said that it was carried out frequently, 18.42% of the students said that it was carried out occasionally, 23.68% of the students said that it was basically not carried out, and 52.63% of the students said that it has never been carried out. The survey data shows that most students are not very familiar with PBL, and PBL has not been carried out in the course. Through the analysis of the students' questionnaire, it was found that their interest in PBL was 15.79% of the students expressed that they were very interested in PBL; 60.53% of the students expressed their interest in PBL; 21.05% of the students expressed that they did not care about PBL. Attitude; 2.63% of students said they are not interested in PBL at all.

The article "Reform of PBL Teaching Mode of Microcomputer System and Embedded Application Course Group" was retracted in 2023. Reasons: signs of a paper mill; suspected computer-generated content; unreliable results or conclusions; concerns about the data.

### 4.2. PBL Teaching Effect Analysis of Microcomputer System and Embedded Teaching Application Group

This experiment conducted a pretest questionnaire and a posttest questionnaire on the help of PBL teaching activities of the microcomputer system and embedded application course group in the form of a questionnaire. In order to ensure the authenticity and validity of the questionnaire results, students were arranged to fill in two questionnaires with similar content before and after the experimental teaching, and they were compared. In the pretest questionnaire, 44.74% of the students said that PBL may not necessarily promote learning; 39.47% of the students said that they did not know; 13.16% of the students said that they could definitely promote; 2.63% of the students said that they could not, as shown in Table 3 and Figure 5 shown.

It can be seen from the statistical results of the questionnaire that in the pretest, because students did not know PBL very well, their attitude towards PBL to promote learning was not very optimistic. Only about 13% of students said that they could promote, and about 84% of students said that Unknown or uncertain attitude. In the posttest questionnaire, after PBL teaching activities, the number of students who said “very effective” and “basically effective” increased significantly.

After the teaching activities, the students' abilities have been improved to varying degrees. In the questionnaire, what gains did PBL bring to you? Among them, 34.38% of the students think that they have gained the ability to collaborate and communicate with others; 25.56% of the students think Learned how to research; 18.75% of the students said that they had acquired professional-related knowledge and experienced the joy of learning; only 1.56% of the students thought there was little gain, as shown in Table 4 and Figure 6. It shows that students have improved their abilities in teaching activities and gained a lot.

The article "Reform of PBL Teaching Mode of Microcomputer System and Embedded Application Course Group" was retracted in 2023. Reasons: signs of a paper mill; suspected computer-generated content; unreliable results or conclusions; concerns about the data.

The PBL mode is used for teaching, which is an experimental class; the traditional teaching mode is used for teaching as a control class. The academic performance evaluation is divided into four evaluation levels of “excellent, good, moderate, and poor,” of which 100–90 is excellent, 89–75 is good, 74–60 is medium, and 59 is poor. The final score is 100 points. From the data in Table 5 and Figure 7, it can be seen that the final academic performance of experimental class students is higher than that of ordinary class.

### 4.3. PBL Teaching Reform of Microcomputer System and Embedded Teaching Curriculum Group

It can be seen from Table 6 and Figure 8 that in the questionnaire on the use of learning resources in PBL teaching activities, 23% of students indicated that they used electronic documents, 22% of students used online teaching courses, and 18% of students used online teaching courses. Using online discussion and communication, 13% of students visited related sites on the Internet. This shows that the computer system has enriched the learning methods of students.

It can be seen from Table 7 and Figure 9 that 32.81% of the students in the questionnaire that think that the main problems of the PBL teaching model exist in the learning process said that the time to complete the task is tight, and 25% of the students said that they need high learning conditions, 17.19% Of the students said that the learning task is difficult, 15.62% of the students said that the efficiency of learning knowledge is low, and 9.38% of the students said that they have high requirements for teachers and students. Students have just come into contact with the PBL teaching model, and their problem awareness and problem inquiry ability have not been established quickly. This is also the most difficult problem students encounter. Therefore, in the process of reforming the PBL teaching model, it is necessary to fully consider the students' learning situation and proceed slowly.

## 5. Conclusion

This article mainly studies the PBL teaching mode reform of the microcomputer system and embedded application course group. This article uses a variety of methods such as literature data method, fuzzy comprehensive analysis method, questionnaire survey method, comprehensive evaluation method to discuss the research theme of this article. Through in-depth study and study of related theories such as microcomputer system and embedded application, PBL teaching mode, design PBL teaching experiment based on microcomputer system and embedded application course group, and compare the effect of teaching experiment.

The article "Reform of PBL Teaching Mode of Microcomputer System and Embedded Application Course Group" was retracted in 2023. Reasons: signs of a paper mill; suspected computer-generated content; unreliable results or conclusions; concerns about the data.

The purpose of this paper is to promote the reform of PBL teaching mode with the aid of computer system and embedded applications. The PBL teaching model can improve students' independent inquiry ability, enhance their interest in learning, and can experience more learning fun in the process of communication and collaboration among students.

The shortcomings of this article are the following points. Firstly, the pace of course implementation is not well controlled, which causes the students to have a tight time to complete the tasks. Secondly, the student grouping should be more subdivided or rationalized. Personality and other aspects are considered; third, due to time and conditions, the sample size of the study is too small, and further research and discussion are needed. PBL teaching practice research is a long-term and meaningful work. It is hoped that the research in this article can better promote the implementation of teaching mode reform.

## Figures and Tables

**Figure 1:** PBL teaching classroom.

**Figure 2:** Basic flow chart of PBL teaching mode.

**Figure 3:** Research status of PBL teaching model in China.

**Figure 4:** Students' understanding and familiarity with PBL.

**Figure 5:** The effect of PBL teaching activities of computer system and embedded teaching application group.

**Figure 6:** Teaching results after the reform of PBL teaching mode.

**Figure 7:** Comparison of experimental results.

**Figure 8:** Information technology support for PBL.

**Figure 9:** Students' problems with PBL teaching.

**Table 1:** Research status of PBL teaching model in China.

Years	Number of related literature	Growth ratio
2008	53	—
2009	97	45.36
2010	98	1.32
2011	143	31.46
2012	173	17.34
2013	178	2.80
2014	217	17.97
2015	215	−0.93
2016	245	12.24
2017	235	−4.25
2018	267	11.98

**Table 2:** Students' understanding and familiarity with PBL.

Subject/knowledge of PBL	Never heard of that	Know a little	To understanding	Know well
Student	71.95	21.34	5.58	3.12
Subject/whether PBL has been carried out	Never started	Basically not started	Occasionally	Often carry out
Student	53.46	24.52	18.11	5.13
Subject/level of interest in PBL	Not interested at all	Doesn't matter	A little interested	Very interested
Student	3.34	21.34	60.28	16.58

**Table 3:** The effect of PBL teaching activities of computer system and embedded teaching application group.

Degree	No effect	Little effect	Basically effective	Very effective
Student's attitude towards PBL to promote learning	3.18	6.65	77.34	14.58
Degree	No	Do not know	Not necessarily	Must be able to
Attitude that can help the course	3.29	39.58	45.52	13.13

The article "Reform of PBL Teaching Mode of Microcomputer System and Embedded Application Course Group" was retracted in 2023. Reasons: signs of a paper mill; suspected computer-generated content; unreliable results or conclusions; concerns about the data.

**Table 4:** Teaching results after the reform of PBL teaching mode.

Teaching function	No effect	Little effect	Basically effective	Very effective
No gain	1.15	2.58	35.58	45.29
Gained professional knowledge	3.32	5.56	25.19	49.76
The ability to collaborate and communicate with others	1.19	5.29	35.78	36.92
Learned how to research	0.28	4.38	34.67	45.29
Experience the joy of learning	0.33	3.29	28.76	55.67

**Table 5:** Comparison of experimental results.

Class	Number of people	Final assessment				The average score	Passing rate
		Excellent	Good	Middle	Bad		
Experimental class	42	2	25	13	2	74.76	95.13
Control class	40	1	16	15	4	70.21	92.30

**Table 6:** Information technology support for PBL.

Education resources	Number of people	Percentage
Multimedia teaching CD	4	3.95
Textbooks and other written materials	17	20.52
Electronic document	19	23.09
Online teaching courses	18	21.79
Online discussion and exchange	15	17.96
Visit related sites on the internet	11	12.83

**Table 7:** Students' problems with PBL teaching.

Problem	Number of people	Percentage	*T* value
Low learning efficiency	11	15.63	3.18
Time to complete the task is tight	22	32.82	2.56
Difficult learning task	11	17.19	3.36
High learning conditions required	17	25.01	3.95
High requirements for teachers and students	7	9.29	4.17
Poor computer performance	13	25.11	4.61
Don't know how to determine the problem	15	29.18	5.26
Don't know how to conduct research	19	37.52	5.24

## Data Availability

No data were used to support this study.

## References

[1] Alrahlah A. (2016). How effective the problem-based learning (PBL) in dental education. A critical review. *The Saudi Dental Journal*.

[2] Rodriguez-Sanchez M. C., Torrado-Carvajal A., Vaquero J., Borromeo S., Hernandez-Tamames J. A. (2016). An embedded systems course for engineering students using open-source platforms in wireless scenarios. *IEEE Transactions on Education*.

[3] Osamnia M., Okada H., Berena A. J., Ueno H., Chunwijitra S. (2016). A novel automated course generation system embedded in the online lecturing platform for higher education. *Computer Applications in Engineering Education*.

[4] Banks R. F., Tiana-Alsina J., Maria Baldasano J. (2016). Sensitivity of boundary-layer variables to PBL schemes in the WRF model based on surface meteorological observations, lidar, and radiosondes during the HygrA-CD campaign. *Atmospheric Research*.

[5] Paredescurin C. R. . (2016). Problem-based learning (PBL): a teaching strategy of environmental education, in cañete municipal school students. *Archives of Surgery*.

The article "Reform of PBL Teaching Mode of Microcomputer System and Embedded Application Course Group" was retracted in 2023. Reasons: signs of a paper mill; suspected computer-generated content; unreliable results or conclusions; concerns about the data.

[6] Diemers A. D, Van d W. M. W. J, Scherpbier A. J. J. A, Baarveld F., Dolmans D. H. J. M. (2016). Diagnostic reasoning and underlying knowledge of students with preclinical patient contacts in PBL. *Medical Education*.

[7] Suciyati H., Hardiansyah (2020). Penggunaan model PBL untuk meningkatkan kemampuan pemecahan masalah matematika dan self efficacy siswa. *JURNAL PENDIDIKAN MIPA*.

[8] Wang T, Liang L, Zheng M. H (2020). Application of formative evaluation and teaching feedback in PBL teaching of Medical Genetics. *Yi chuan = Hereditas*.

[9] Noor N. A. M., Saim N. M., Alias R., Rosli S. H. (2020). Students’ performance on cognitive, psychomotor and affective domain in the course outcome for embedded course. *Universal Journal of Educational Research*.

[10] Kim H. K. (2016). Course-embedded assessment in Korean nursing baccalaureate education. *Korean Journal of Medical Education*.

[11] Coppock P., Park S. H., Paredes J. (2017). Enhancing research skills and attitudes in undergraduate organic chemistry with a course-embedded undergraduate research experience (CURE) via green organic synthesis. *Journal of Laboratory Chemical Education*.

[12] Larson J, Jordan S. S, Lande M, Weiner S. (2020). Supporting self-directed learning in a project-based embedded systems design course. *IEEE Transactions on Education*.

[13] Üstünel H. (2020). A project based innovative approach to an embedded systems course laboratory in software engineering education. *Computer Applications in Engineering Education*.

[14] Nam S. M., Mi (2017). Development of a program outcomes assessment system based on course embedded assessment for nursing education. *The Journal of Korean Academic Society of Nursing Education*.

[15] Fic C. (2018). Working as an embedded archivist in an undergraduate course: transforming students into scholars through an archival workshop series. *American Archivist*.

[16] Westera W., Verpoorten D. (2016). Structured reflection breaks embedded in an online course - effects on learning experience, time on task and performance. *Interactive Learning Environments*.

[17] Fernandes M. A. (2016). Project-based learning applied to an embedded systems course. *International Journal of Electrical Engineering Education*.

[18] Chung J, Hak K. C (2016). Development and implementation of design tool for course-embedded assessment in the engineering education accreditation. *Journal of Engineering Education Research*.

[19] Lei Y. . (2018). Design and implementation of a new wireless remote control cipher lock system based on single chip microcomputer. *International Journal for Engineering Modelling*.

[20] Perovich D. K., Hirai A. (2017). Microcomputer-based image-processing system. *Journal of Glaciology*.

The article "Reform of PBL Teaching Mode of Microcomputer System and Embedded Application Course Group" was retracted in 2023. Reasons: signs of a paper mill; suspected computer-generated content; unreliable results or conclusions; concerns about the data.

[21] Mcneil B., Díaz J. C., Bruns C. (2018). Determining the time required to detect induced sow lameness using an embedded microcomputer-based force plate system. *American Journal of Animal and Veterinary Sciences*.

[22] Akgul A, Yldz M. Z, Boyraz M. F (2020). Microcomputer-based encryption of vein images with a nonlinear novel system. *Journal of the Faculty of Engineering and Architecture of Gazi University*.

[23] Tech Res Inst (2017). The interactive design system based on a microcomputer for prevention works of landslide. *Geological data processing*.

